# Evidence for the Role of Mindfulness in Cancer: Benefits and Techniques

**DOI:** 10.7759/cureus.4629

**Published:** 2019-05-09

**Authors:** Ria Mehta, Kirti Sharma, Louis Potters, A. Gabriella Wernicke, Bhupesh Parashar

**Affiliations:** 1 Radiation Medicine, Zucker School of Medicine at Hofstra / Northwell, New York, USA; 2 Radiation Oncology, Zucker School of Medicine at Hofstra / Northwell, New York, USA; 3 Radiation Oncology, NewYork-Presbyterian/Weill Cornell Medical Center, New York, USA

**Keywords:** mindfulness, cancer, stress, fatigue, pain, techniques

## Abstract

Mindfulness is being used increasingly in various aspects of cancer management. Benefits of mindfulness practices are being observed to manage the adverse effects of treatment, symptoms from cancer progression, and the cost-effectiveness compared to conventional contemporary management strategies. In this review article, we present clinical trial data showing the benefits of mindfulness in various aspects of cancer management as well as techniques that have been commonly used in this practice.

## Introduction and background

The definition of mindfulness as stated by Merriam-Webster is as follows: (a) The quality or state of being mindful and (b) The practice of maintaining a nonjudgmental state of heightened or complete awareness of one's thoughts, emotions, or experiences on a moment-to-moment basis. 

Mindfulness-based meditations originated from ancient Eastern religious traditions such as Hinduism and Buddhism. The current approach to mindfulness, as understood in the Western health system, is a way to achieve a state of mind that is aware and in control. This approach, in turn, reduces stress, improves physical health, and allows harmony in life. There are other mindfulness practices in existence but they may be secretive and not discussed in public.

However, in the Eastern philosophies, approach to mindfulness is somewhat different. It is a set of techniques to achieve a state of mind that is used to experience higher awareness or consciousness. Mindfulness has also been described in ancient literature to enhance physical and mental wellbeing. This may be helpful for cancer patients [1]. The diagnosis of cancer and its treatment-related toxicity causes severe emotional distress in patients and their caregivers [2]. Unfortunately, pharmacological interventions used to alleviate the adverse symptoms are also associated with their own undesirable side effects. Therefore, there is a need to develop non-pharmacologic interventions to deal with these adverse effects. In this review, we discuss evidence of the utility of mindfulness in cancer management.

## Review

Methods

We performed a PubMed search on ‘mindfulness’ and ‘cancer’ and selected ‘clinical trials’ as a filter. Search results yielded 124 studies from 2000-2018. Studies were selected for review if it addressed one of the following aspects of cancer management: cancer prevention, cancer-related stress, cancer-related pain, cancer-related fatigue, cancer-related cachexia, cancer-related sleep disorders, immune response and mindfulness, caregivers of cancer patients, radiation therapy, and cost-effectiveness. In the end, we describe some mindfulness techniques that have been described and whose adaptations have been used in cancer.

A potential benefit of mindfulness on cancer prevention

In a hypothesis-generating study, a prospective study measured and compared 12-hour urinary 6-sulfatoxymelatonin between women who regularly meditated versus those who did not. Women in the meditation group had increased levels of physiological melatonin compared to the non-meditation group. This is significant since melatonin has been shown in multiple studies to have anti-cancer properties [3,4] as well as other biologic functions important in maintaining health and preventing disease such as immunomodulation and hematopoiesis [4].

Mindfulness and cancer-related stress

Diagnosis of cancer is a highly stressful event. It is commonly associated with depression (prevalence 5%-15%) and has been shown to increase the number of suicides [5, 6]. Mindfulness has been evaluated in a number of studies in the management of cancer-related depression and stress.

In a study to determine the efficacy of a Mindfulness-Based Stress Reduction (MBSR) intervention for mood disorders in women with breast cancer (BC), a randomized controlled trial (RCT) assigned 166 women to the MBSR group versus non-MBSR groups [7]. This was a five-year longitudinal randomized trial in women who had completed breast cancer treatment including chemotherapy/hormones and radiation therapy. MBSR included either eight-week self-instructing sessions with or without an instructor, weekly group sessions or no intervention. Mood disorders were measured using the Hospital Anxiety and Depression (HAD) Scale, which is a 14-item questionnaire measuring anxiety and depression. Other scales that were used in the assessment were Memorial Symptom Assessment Scale (MSAS), 36-item Short Form Health Survey (SF-36), Sense of Coherence scale (SOC), Five Facets of Mindfulness Questionnaire (FFMQ-Swedish version), Post-Traumatic Growth Inventory (PTGI), lymphocyte distribution, NK-cell activity, and cytokine levels. Women in the MBSR group experienced significant improvements in depression scores, physical and psychological measures, and better-coping capacity. The mean pre-MBSR HAD score was 4.3 and post-MBSR score 3.3 (p = 0.001) compared to non-MBSR (p = 0.015). There was a significant increase in the NK-cell activity in the MBSR group, changes in the lymphocyte counts but no changes in cytokine levels in the two groups. Scores for distress, symptom burden, immune response, and mental health also showed significant improvements.

To study the efficacy of the Cognitively-Based Compassion Training (CBCT) in BC patients, an RCT randomly assigned participants to CBCT or a Treatment-As-Usual (TAU) control group [8]. Participants were adults with a history of BC in the last 15 years but cancer free at the time of the study, on no active treatment. CBCT is based on Tibetan Buddhist meditative techniques and in this study was composed of eight-week consecutive sessions. CBCT is different from Mindfulness-Based Interventions (MBI) because it involves an analytical and cognitive approach to mindfulness. MBI practices involve a non-judgmental stance towards emotions and practices. Measures included Functional Assessment of Cancer Therapy-Breast Cancer (FACT-BC), physical quality of life (QoL), emotional and functional QoL, Brief Symptom Inventory (BSI-18), Fear of Cancer Recurrence Inventory (FCRI), Self-Compassion Scale short form, and FFMQ-short form. The final number of participants was 56. A within-group comparison showed a significant improvement in pre-to-post CBCT intervention versus no significant change in the TAU group with respect to self-kindness, self-judgment, common humanity, over-identification, mindful observation, acting with awareness skillsets and self-compassion. CBCT was effective in diminishing stress caused by fear of cancer recurrence (FCR).

A prospective study in adult patients with any cancer diagnosis, early stage or recurrent cancer except brain cancer, assessed the outcomes of an eight-week Mindfulness-Based Art Therapy (MBAT) intervention [9]. MBAT involves the practice of opening to artist-grade art media, making a collage using various techniques, use of digital photography away from the medical facility for four to five of the eight-week program. The process is meant to enhance intrapersonal meaning with non-verbal creative expression. MBAT is a combination of MBSR and art therapy programs and is meant to reduce negative association with illness. Walkabout: Looking In, Looking Out, a part of the MBAT program combines MBSR and art therapy program. Measures in this study included Edmonton Symptom Assessment Scale R (ESAS-R) for symptoms by cancer patients, Pittsburgh Sleep Quality Index (PSQI), SF-36, Antonovsky’s Sense of Coherence Orientation of Life Questionnaire-29 for symptoms experienced, and Functional Assessment of Chronic Illness Therapy-Spiritual Wellbeing (FACIT-SP). MABT intervention (n=18) resulted in significant improvement in depression, sense of coherence, health-related QoL, and on spiritual well-being.

In an RCT to assess the MBSR program on mood disturbance and symptoms of stress in cancer out-patients (all patients with a diagnosis of cancer eligible), participants were assigned randomly to either an immediate treatment condition or a wait-list control condition [10]. The MBSR program was based on the one devised by Kabat Zinn [11]. The program consists of three parts: theory, meditative and yoga practices, group processes focused on problem-solving. The primary outcomes were measured using the Profile of Mood States (POMS) and Symptoms of Stress Inventory (SOSI). Post-intervention scores were calculated until the six-month follow-up. Eighty-nine patients were enrolled in the trial. There was a significant reduction in POMS score suggesting a reduction in mood disturbance with intervention. There was also a significant reduction in the subscales of mood disturbance post-intervention: anger, anxiety, depression, and confusion. SOSI scores showed a significant reduction post-intervention, which represents a reduction in stress. Post-subscales such as cardiopulmonary, depression, emotional irritability, cognitive disorganization, muscle tension, and gastrointestinal symptoms also showed a significant reduction. The overall reduction in total mood disturbance was 65% with a 31% reduction in symptoms of stress.

A study evaluated the impact of a theoretical-empirical based intervention (ConquerFear) on FCR [12]. Participants were patients with breast cancer, colorectal cancer, or melanoma. Patients had completed the curative treatment two months to five years prior to study enrollment and were cancer free at the time of accrual. ConquerFear is a manualized intervention that uses strategies to overcome excessive fear, modify unhelpful beliefs and worry, and develop behavior to reduce the risk of recurrence. The attention control, ‘taking it easy’, involves meditative techniques, visualization, and quick-relaxation techniques. The primary outcome measure in the study was a 42-item FCRI. Other measures included FCRI subscales, a 22-item Impact of Event Scale (IES) revised, a 21-item DASS21 (21 item Depression Anxiety Stress Scale), a 35-item assessment of quality of life (AQoL8D), a 30-item metacognition questionnaire (MCQ30), survivors unmet need survey, and a six-item credibility/expectancy questionnaire. Participants were randomized to 1:1 ratio to either five face-to-face sessions of ConquerFear or attention control “taking-it-easy’ group. The total FCRI scores decreased significantly in the ‘ConquerFear’ group versus the ‘taking-it-easy’ participants, showing a positive impact of the ConquerFear intervention. This was also true of all FCRI subscales. ConquerFear also had significantly better outcomes with regards to general anxiety, cancer-specific anxiety, mental health, and overall QoL.

In a large RCT to evaluate the efficacy of the MBSR (BC) program compared to usual care (UC) in normalizing blood levels of pro-inflammatory cytokines among BC survivors (BCS), 322 patients with stage 0-III BC survivors were recruited [13]. This MBSR was based on Kabat-Zinn techniques [11]. It consists of sitting meditation, body scan, gentle hatha yoga, walking meditation, and informal practice. Curative treatments should have been completed within two weeks to two years prior to study enrollment. Patients were randomized to either a six-week MBSR(BC) program or a UC program. At baseline and six and twelve weeks, blood samples were collected and assessed for plasma cytokines (interleukin [IL]-1β, IL-6, IL-10, tumor necrosis factor [TNF] α, transforming growth factor [TGF] β1, soluble tumor necrosis factor receptor [sTNFR] 1). TNFα and IL-6 increased during the follow-up period at a higher rate during the MBSR(BC) training period versus the UC group, while sTNFR1 levels did not change significantly across the 12-week period. The authors commented that increases in TNFα and IL-6 were markers for immune restoration, thereby showing the beneficial effects of MBSR.

An RTC was performed to test mindfulness meditation practice, when delivered during one session of active chemotherapy administration, on the acute salivary cortisol (a marker of neuroendocrine system activity) in cancer patients [14]. Fifty-seven patients were enrolled in the trial. Eligible patients were adults with colorectal cancer (CRC), about to begin chemotherapy. Patients were blinded into one of the three groups in 1:1:1 ratio; standard chemotherapy group versus cancer education module group or a mindfulness group plus cancer education module group. Mindfulness practice was a pre-recorded audiovisual instruction on guided mindful meditation. Saliva cortisol reflects physiologically active free cortisol. Behavioral measures included Multidimensional Fatigue Symptom Inventory (MFSI), DASS, and Mindfulness Attention Awareness Scale (MAAS). Saliva samples were collected at the start of chemotherapy and at subsequent 20-minute intervals during the first 60 minutes of chemotherapy. More than twice as many patients in the mindfulness group versus the controls showed a cortisol rise suggesting that mindfulness practice during chemotherapy can reduce the hypothalamic pituitary axis (HPA) blunting profiles typically observed in cancer patients. MAAS significantly anti-correlated with MFSI and DASS while MFSI correlated with DASS.

Supportive-Expressive Therapy (SET) is based on the idea that patients' capacity to cope with their cancer is improved by expressing their emotions and increasing their social support. MBCR (Mindfulness-Based Cancer Recovery) is the MBSR program adapted for cancer patients and their recovery. In a study comparing MBCR versus SET in BC survivors, 252 patients were enrolled in the study. The measures included the Profile of Mood States (POMS), a 56-item Calgary Symptoms of Stress Inventory (CSOSI), FACT-B, Medical Outcomes Study Social Support Survey (MOS-SSS) and MAAS. MBCR in distressed BC survivors was found to be superior to SET for improving psychological well-being with benefits lasting over a year compared to controls [15,16].

In patients with low-risk prostate cancer placed on active surveillance, researchers conducted a feasibility and preliminary efficacy study of an eight-week MBSR session. The participants were randomized to either MBSR (n = 24) or an attention control arm (n = 19). Participants in the control group received a book on mindfulness called ‘Full Catastrophe Living’ with no specific instructions to read it. Participants in the mindfulness arm participated in the eight-week intervention done by a trained instructor. The measures used in this study included the Memorial Anxiety Scale for Prostate Cancer (MAXPC), Post-Traumatic Growth Inventory (PTGI), Intolerance of Uncertainty Short Form (IUS), MAAS, and PROMIS-Global Health 10 (PGH-10). Mindfulness intervention demonstrated significant decreases in prostate cancer anxiety and uncertainty intolerance, and significant increases in mindfulness, global mental health and post-traumatic growth [17].

A randomized control trial in Chinese patients with BC showed improvements in post-traumatic growth (PTG) and Perceived Stress Scale of Chinese version (CPSS) in the MBSR group with results that persisted three months after intervention [18]. In another study in Danish women with BC, benefits of MBSR were seen on somatic symptoms that stayed for six months after intervention [19].

In an RCT in premenopausal women with BC, women were randomly assigned to a six-week Mindful Awareness Practices (MAPs) intervention group or to a wait-list control group. MAPs is a six weekly two-hour session theory on mindfulness, practice of meditation and gentle movement exercises, lectures, discussions, and group practices as well as home practice sessions. MAPS intervention led to reductions in perceived stress, reductions in depressive symptoms as well as reductions in proinflammatory gene expression and inflammatory signaling [20]. In an RCT in BC patients evaluating MBSR and SET on telomere length (TL), TL in the intervention group was maintained whereas it was found to decrease for control participants. TL has been shown to decrease under stress [21].

The Contemplative Self-Healing program is a 20-week meditation-based stress reduction program, which consists of eight weekly 90-minute sessions on teaching meditation skills. Exercises include awareness of breath, healing imagery, and deep breathing. In a pilot project to evaluate the QoL outcomes of a 20-week contemplative self-healing program, women with a history of stage I-III BC were assessed using FACT- G, FACT-B, Functional Assessment of Chronic Illness Therapy-Spirituality (FACIT-Spirituality), ECOG, and the Impact of Events Scale. Intervention showed improved QoL with a clinically and statistically significant increase in the FACT-G and a significant reduction in post-traumatic stress symptoms assessed by the Impact of Events Scale [22].

Mindfulness and cancer-related pain

Pain occurs in 20% to 50% of patients with cancer, and approximately 80% of patients with advanced-stage cancer have moderate to severe pain [23, 24]. Current management techniques commonly used include medications, radiation therapy, chemotherapy, agents used as nerve blocks, radioisotopes. Mindfulness has recently been explored as an effective pain control modality.

MBCT showed a statistically significant, robust, and durable effect on pain intensity in 129 women with BC randomly assigned to an eight-week MBCT program versus a wait-list control group. The measures used included short-form McGill Pain Questionnaire-2 (SF-MPQ-2), the Present Pain Intensity Subscale (the PPI of the McGill Pain Questionnaire) and Numeric Rating Scales, World Health Organization-5 Well-Being Index, Hospital Anxiety and Depression Scale, and self-reported use of pain medication. The intervention resulted in statistically significant improvement in pain intensity. Statistically significant effects were also observed for QoL and nonprescription pain medication use [25].

Mindfulness and cancer-related fatigue (CRF)

A recent study found a prevalence of 45% of moderate to severe CRF in cancer survivors [26], which is a major cause of distress in cancer survivors [27]. We summarize some of the recent studies exploring mindfulness to manage CRF. In a prospective RCT [28-30], BC and CRC survivors with moderate-to-severe fatigue were randomized to MBSR or a fatigue Education and Support (ES) condition. Measures utilized were Attentional Function Index (AFI) and the Stroop test. MBSR participants reported significantly greater improvement on the AFI total score and greater Stroop accuracy rates compared to ES participants [29].

Mindfulness and cancer-related cachexia

An important study in various Eastern Cooperative Oncology Group (ECOG) chemotherapy trials reported that the greatest incidence of weight loss was seen among patients with solid tumors [31]. About 50% of prostate, colon, and lung cancer patients and 85% of gastric/pancreatic patients lost weight, while 30% of those with BC or acute leukemia had weight loss. One-third had more than 10% weight loss, although any weight loss (0%-5%) was associated with a poorer prognosis when compared to patients with no weight loss. Cancer cachexia is defined as a multifactorial syndrome defined by an ongoing loss of skeletal muscle mass that leads to progressive functional impairment. Its pathophysiology is characterized by a negative protein and energy balance driven by a variable combination of reduced food intake and abnormal metabolism. Diagnostic criterion for cachexia is weight loss greater than five percent, or weight loss greater than two percent in individuals already showing depletion according to current bodyweight and height (body-mass index [BMI] <20 kg/m(2)) or skeletal muscle mass (sarcopenia) [32]. Mindfulness has been studied to counter this distressing symptom.

Subjects developing cachexia symptoms while being treated for cancer were randomized in an RCT aiming to compare an experimental group that would participate in specific workshops based on mindfulness alternating dietetic and psychological approaches, and a control group managed in accordance to usual practice. Recruitment was difficult (12% of the approached population). Eventually, 53 patients participated. This study used mindfulness workshops that included four double workshops every two weeks. In the diet workshops, food was tested through five senses. Enrichment techniques and tasting of particular dishes were developed. In comparison with the control group, patients randomized to the experimental group showed a significant benefit with an increase in their body weight and an improvement of their World Health Organization (WHO) status score. They also experienced an improvement in emotional function and observation faculty as well as a relief of fatigue and some digestive disorders [33].

Cancer-related sleep disorders

Sleep disturbances are commonly experienced by patients with cancer. Patients describe problems falling asleep (sleep latency), problems staying asleep (awakenings), having restless sleep (quality of perceived sleep), and/or having trouble staying awake during the day (excessive daytime sleepiness). The issues of sleep-wake disturbances are often combined with cancer-related fatigue and insomnia, which occur pretreatment, exacerbate during treatment, and continue through survivorship [34]. Mindfulness has been studied for sleep benefit in cancer patients and survivors.

A study investigated MBSR versus UC for BC survivors on multiple measures of subjective sleep. The measures used included subjective sleep parameters (SSP), Pittsburgh Sleep Quality Index (PSQI) and objective sleep parameters (OSP). Results showed a positive effect of MBSR on OSP, percent of sleep time, and less number waking bouts [35].

In a secondary analysis of an RCT comparing MBCR to Cognitive Behavior Therapy for Insomnia (CBT-I) in cancer patients, changes in dysfunctional sleep beliefs produced by the CBT-I group exceeded those produced by MBCR at post-program and follow-up. However, there were no significant differences between the groups in patients exceeding insomnia severity [36].

In an RCT [37], investigators evaluated the effects of two mind-body interactions, mind-body bridging (MBB) and mindfulness meditation (MM) versus sleep hygiene education (SHE) control on salivary oxytocin (SOT) levels in cancer survivors. MM included basic meditation techniques, body scans, walking meditation, and forgiveness meditation. MBB teaches mindfulness and awareness skills to help become aware of potentially dysfunctional mental and bodily states, and individuals are taught to pay attention to sights, sounds, sensations to calm their mind and relax the body. In SHE, instructors discuss various sleep topics with the participants such as causes of sleep disturbance, worries, concerns as well as tips to improve sleep. Oxytocin is a neuropeptide hormone that is involved in a number of human physical and psychosocial processes such as labor, social bonding, altruism, cooperation, wellbeing, to name a few. This study was an exploratory study to assess the effects of various mindfulness-based interventions on SOTs. Other outcome measures included MOSS, PSS (Perceived Stress Scale), Center for Epidemiological Studies -Depression Scale (CES-DS), FACT-G, Well-Being Index (WBI), Five-Facet Mindfulness Questionnaire (FFMQ), and Self-Compassion Scale (SCS). SOT levels were significantly greater post-intervention in MBB compared to SHE but did not differ between SHE and MM. Greater reductions in sleep problems were noted for MBB and MM compared with that of SHE and increases in mindfulness and self-compassion were observed in the MBB group compared with those in SHE (37). An RCT conducted in Calgary, Alberta, Canada compared MBSR to CBT-I for the treatment of insomnia. MBSR was inferior to CBT-I for improving insomnia severity immediately after the program but MBSR demonstrated non-inferiority at follow-up [38].

In another study to assess MBSR in BC patients on sleep quality, mean sleep problem scores were significantly lower in the MBSR group than in controls immediately after the intervention. After the 12-month follow-up, there was no significant between-group effect of MBSR on sleep quality in intention-to-treat analyses [39].

Mindfulness during radiation therapy

The relative effectiveness of MBSR compared to a Nutrition Education Program (NEP) and UC in women with early-stage BC undergoing radiotherapy (RT) was tested, and the women who actively received radiotherapy (ART) while participating in the MBSR intervention (MBSR-ART) experienced a significant improvement in multiple psychosocial variables compared with the NEP-ART, UC-ART, or both at four months [40].

Mindfulness and immune response

The role of mindfulness in modulating immune response has been studied. In an RCT conducted to examine immune recovery following BC therapy and evaluation of MBSR on immune recovery, patients were randomized into an MBSR versus UC group. Women in the MBSR group had T cells more readily activated by the mitogen phytohemagglutinin (PHA) and an increase in the Th1/Th2 ratio. MBSR also promoted a more rapid recovery of functional T cells capable of being activated by a mitogen with the Th1 phenotype, whereas substantial recovery of B and NK cells after completion of cancer treatment appeared to occur independently of stress-reducing interventions [41]. Other studies have shown an improvement in increased NK cell cytolytic activity post-MBSR [42, 43].

Mindfulness for caregivers of cancer patients

Cancer is truly a disease that afflicts not just the patients but the entire family or caregivers. The stress and pain that the patients suffer are experienced to a significant extent by the patient’s family and/or caregivers. Mindfulness can potentially be useful for the support team of patients suffering from cancer.

In a study to explore the effects of a mindfulness intervention to cultivate patient and caregiver capacity to respond to the challenges of cancer with greater ease, the Mindfully Optimizing Delivery of End-of-Life (MODEL) Care intervention was used. MODEL Care intervention enhanced patient and caregiver capacity to respond to the emotional challenges that often accompany advanced cancer and decreased patient and caregiver psychological barriers to advanced care planning [44]. However, another RCT that evaluated MBSR versus UC in lung cancer patients failed to show a positive impact on caregivers although the significant benefit of intervention was noted in patients [45].

Cost-effectiveness

Several studies have shown mindfulness interventions to be more cost-effective compared to traditional approaches to manage stress and QoL outcomes. In a study examining the cost-effectiveness of MBSR on BC survivors, cost per quality-adjusted life year was relatively low compared to the cost-utility findings of other published BC interventions and it appeared to provide an improved health-related QoL at a comparatively low cost [46]. However, in another study evaluating MBAT program versus BC Support Group (BCSG) for cost-effectiveness, the overall cost for 191 participants in the MBAT intervention group was $992.49 per participant compared with $562.71 per participant for the BCSG intervention. Although the MBAT intervention was more costly, sensitivity analysis showed that the cost-effectiveness of the MBAT intervention could achieve parity with that of a BCSG if some intervention-related costs, such as staff time and supplies, were reduced [47].

When cost-effectiveness of MBCT was compared to a wait-list control group for pain in women with BC, the primary outcome was the Minimal Clinically Important Difference (MCID) on pain intensity. The MBCT was cost-effective with a probability of 85%, and additional women achieving MCID set to zero remained cost-effective with a probability of 70% to 82% when smaller effect and higher MBCT costs were assumed [48].

A summary of seminal studies and their outcomes is listed in Table 1.

**Table 1:** Summary of seminal studies showing effects of mindfulness-based techniques on cancer patients Abbreviations: NA - Not Applicable, MBSR - Mindfulness-Based Stress Reduction, CBCT - Cognitively-Based Compassion Training, MBAT - Mindfulness-Based Art Therapy, CRC - Colorectal Cancer, MAPS -Mindful Awareness Practices, MBCT - Mindfulness-Based Cognitive Therapy, PES - Psychoeducation Support, MBCR - Mindfulness-Based Cancer Recovery, MBB - Mind-Body Bridging, MM - Mindfulness Meditation, MODEL - Mindfully Optimizing Delivery of End-of-Life, NK - Natural Killer (cells)

Study reference no.	Cancer type	Mindfulness technique	Benefits (statistically significant)	Outcomes/comments
3	Breast cancer	urinary 6-sulphatoxymelatonin measured	Meditation beneficial	NA
7	Breast cancer	MBSR	Beneficial	Stress
8	Breast cancer	CBCT	Beneficial	Stress
9	Cancer	MBAT	Beneficial	Stress
10	Cancer	Meditation	Beneficial	Stress
12	Breast/CRC/melanoma	ConquerFear	Beneficial	Stress/anxiety
13	Breast cancer	MBSR	Beneficial	Proinflammatory cytokines
14	CRC	Mindfulness	Beneficial	Blunting of neuroendocrine profiles
15	Breast cancer	MBSR	Beneficial	Wellbeing
17	Prostate cancer	MBSR	Beneficial	Anxiety
18	Breast cancer	MBSR	Beneficial	Stress
19	Breast cancer	MBSR	Beneficial	Stress
20	Breast cancer	MAPS	Beneficial	Stress
21	Breast cancer	MBSR	Beneficial	Stress
22	Breast cancer	Contemplative self -healing	Beneficial	Stress
25	Breast cancer	MBCT	Beneficial	Pain
28	Breast cancer/CRC	MBSR/PES	Beneficial	Fatigue
29	Breast cancer/CRC	MBSR	Beneficial	Fatigue
30	Cancer survivors	MBSR	Beneficial	Fatigue
33	Cancer patients	Mindfulness	Beneficial	Cachexia
35	Breast cancer	MBSR	Beneficial	Sleep
36	Cancer	MBCR	Beneficial	Sleep
37	Cancer survivors	MBB/MM	Beneficial	Sleep
38	Cancer	MBSR	Beneficial	Sleep
39	Breast cancer	MBSR	Beneficial	Sleep
41	Breast cancer	MBSR	Beneficial	T cell function
42	Cancer	MBSR	Beneficial	NK cytolytic activity
43	Breast cancer	MBSR	Beneficial	NK cell activity
44	Cancer	MODEL intervention	Beneficial	Caregivers+patients
45	Lung cancer	MBSR	Not beneficial	Caregivers (although benefited patients)
46	Breast cancer	MBSR	Beneficial	Cost-effective
47	Breast cancer	MBAT	Not beneficial	Cost-effective
48	Breast cancer	MBCT	Beneficial	Cost-effective

Techniques

There are several techniques for practicing mindfulness; however, the primary aim is to bring the mind to focus on either an internal or external entity. Techniques may include the mind focusing on an external gross object, an external or internal sound, or on observing one’s breath. Mindfulness requires practice so that each technique can help the mind to stabilize rather than be active. A comprehensive commentary of origins and techniques of mindfulness is described elsewhere [11, 49], although a brief summary of techniques used is tabulated below (Table 2).

**Table 2:** Common techniques used in MBSR MBSR - Mindfulness-Based Stress Reduction

Technique	Description
Body scan	Patients focus awareness on individual parts of the body.
Sitting meditation	Participants instructed to sit down in a comfortable position and direct their full attention on sensation of breathing.
Mindful Hatha yoga	Yoga stretches and postures with the focus on body awareness rather than form.
Non-judging	A person intentionally pays full attention to whatever is occurring at the current moment without judging it.
Patience	Practice the knowledge that things unfold in their own time.
Beginner’s mind	Practice to see everything as if it were happening for the first time and being present in one’s experience.
Trust	One learns to honor one's own feelings rather than to suppress or distrust them.
Non-striving	Practicing to have no goal other than meditation itself. State of not doing anything, just accepting what comes.
Letting go	Practicing to neither try to hold on to or reject your experience.
Kindness	Understanding one’s difficulties and being kind and warm in the face of difficulties and avoiding being self-critical.
Curiosity	Focus of a person’s attention is opened to admit whatever enters experience, a stance of kindly curiosity allows the person to investigate whatever appears without automatic judgment.
Acceptance	Completely accepting the thoughts, feelings, sensations, and beliefs that one has, and understanding that they are simply those things only.

## Conclusions

Mindfulness-based practices are being increasingly utilized in various aspects of cancer management. It has shown utility in multiple prospective trials and continues to be explored. Most of the evidence of the benefit of mindfulness in cancer is to reduce toxicity and stress. There is a need for more prospective trials exploring its use in reducing cancer incidence or preventing its recurrence.
